The article "Application of Genetically Encoded Molecular Imaging Probes in Tumor Imaging" was published in 2022. Journal: Contrast Media Mol Imaging.

# Application of Genetically Encoded Molecular Imaging Probes in Tumor Imaging

**DOI:** 10.1155/2022/5473244

**Published:** 2022-08-27

**Authors:** Meng Du, Ting Wang, Yaozhang Yang, Fengyi Zeng, Yue Li, Zhiyi Chen

**Affiliations:** ^1^The First Affiliated Hospital,Medical Imaging Centre,Hengyang Medical School, University of South China, Hengyang 421001, Hunan, China; ^2^Institute of Medical Imaging,Hengyang Medical School, University of South China, Hengyang 421001, Hunan, China; ^3^Laboratory of Ultrasound Molecular Imaging, the Third Affiliated Hospital of Guangzhou Medical University, Guangzhou 510000, Guangdong, China

## Abstract

In recent years, imaging technology has made rapid progress to improve the sensitivity of tumor diagnostic. With the development of genetic engineering and synthetic biology, various genetically encoded molecular imaging probes have also been extensively developed. As a biomedical imaging method with excellent detectable sensitivity and spatial resolution, genetically encoded molecular imaging has great application potential in the visualization of cellular and molecular functions during tumor development. Compared to chemosynthetic dyes and nanoparticles with an imaging function, genetically encoded molecular imaging probes can more easily label specific cells or proteins of interest in tumor tissues and have higher stability and tissue contrast *in vivo.* Therefore, genetically encoded molecular imaging probes have attracted increasing attention from researchers in engineering and biomedicine. In this review, we aimed to introduce the genetically encoded molecular imaging probes and further explained their applications in tumor imaging.

## 1. Introduction

Imaging plays an integral role in the diagnosis and treatment of tumors, which makes the process of the occurrence and development of diseases visualized [1]. Currently, there are several imaging methodologies that are widely used in clinical practice, such as X-ray imaging, magnetic resonance imaging (MRI), ultrasonic imaging, and radionuclide imaging. However, due to the limitation of sensitivity and accuracy, the traditional imaging technique can only show the anatomic and functional changes of organs and tissues, which is incapable of early diagnosis of tumors.

Molecular imaging is a newly developed medical imaging method, which allows monitoring of biological processes at both the cellular and subcellular levels [2], realizing the earlier period and noninvasive diagnosis of tumors. Molecular imaging probes are a crucial component for efficient tumor imaging *in vivo* [3, 4]. The chemosynthetic probe is commonly applied in molecular imaging, which consists of two modules. One is an imaging module to provide detectable signals, and the other is a targeting module to bind a specific site of lesion or react specifically with certain molecules. Although those probes demonstrated enhanced imaging visualized at the cell molecular level, it still has biosafety concerns, such as intolerable chemical toxicity [5]. Furthermore, a chemosynthetic probe can only achieve instantaneous imaging rather than longitudinal monitoring.

With the rapid development of genetic engineering technology and synthetic biology, genetically encoded molecular imaging probes have gradually become the research focus of visualization in cancer diagnosis and treatment. Imaging probes (protein) can be continuously produced by genetically encoded molecular probes infecting cells directly or by integrating the image probes genes into the cancer cells' genome, realizing real-time and persistent imaging in tumors (Figure 1). It has shown high sensitivity and spatial resolution imaging signals, and the advantage of great kinetics, metabolic stability, and biocompatibility, which benefits *in vivo* tumor imaging to realize local dynamic monitoring for precise tumor imaging [6], resolving the problems of the abovementioned imaging techniques in spatial and temporal resolution, penetration depth, and timeliness [7, 8].

The imaging protein can be stably expressed, and it can visually observe the change in the primary site of the tumor for predicting the occurrence and development of the tumor. For example, the reporter gene can be transfected or transduced into the tumor cell, which can express specific probes to posttranscriptional modification, protein interactions, and so on. It has been reported that GFP, HSV1TK, and firefly luciferase reporter genes were transfected into the tumor genome to determine the presence of tumor metastasis at the cellular level [9]. At present, it has been reported that various kinds of genetically encoded molecular imaging probes, such as proteins, enzymes, or cell surface receptors, via different imaging methods, have been used for cancer monitoring. These probes can provide visualization space at the molecular or genetic level for tumors [10]. Thus, using probes via genetic engineering is an effective way for precise tumor local imaging.

In this review, we will first introduce the significance of genetically encoded molecular imaging probes in *in vivo* tumor imaging and analyze in detail the application of probes in different imaging modalities. We also mention the obstacles of realizing the clinical transformation of genetically encoded molecular imaging probes. Finally, we briefly discuss the limitations and future of the application of genetically encoded molecular imaging probes in tumor imaging.

## 2. Application of Various Imaging Modalities Based on Genetically Encoded Probes in Tumor Imaging

Recently, specific gene-editing imaging probes used for tumor imaging have been developed and validated in various imaging modalities, including optical imaging, US imaging, MR imaging, and radionuclide imaging. Then, we will introduce using gene-synthesized molecular imaging probes in various imaging modalities for tumor imaging.

### 2.1. Optical Imaging

Optical imaging is a novel imaging method, including bioluminescence imaging, fluorescence imaging (FI), photoacoustic imaging (PAI), and optical tomography. Optical imaging with the advantages of noninvasive and high-resolution features has been applicated for biomedical imaging [11, 12]. At present, optical molecular imaging probes, which can realize the visualization of the structure and function of tumor cells, even at the subcellular level, have been developed [13, 14]. Genetically encoded optical probes, such as fluorescent protein, and luciferase, can label cell membrane, organelle, and even the specific molecules involving tumor metabolism. The most common application is to establish tumor-bearing model with tumor cells encoding luciferase or fluorescent protein, which realizes noninvasive monitoring of tumor volume and tumor metastasis through optical imaging.

#### 2.1.1. Fluorescence Imaging

Imaging combined with a reporter gene, such as the green fluorescence protein (GFP) gene, provides a noninvasive tool for monitoring genetic function. Fluorescent proteins are composed of spectrally distinct proteins, which generally have short emission spectra and high quantum yield. The molecular weight of the fluorescent protein is generally between 25 kDa and 30 kDa, and the fluorescent mainly depends on the chromophore formed inside, not limited by other cofactors. With the wide application of imaging with a fluorescent protein, various fluorescent probes have been designed to realize tumor imaging and even tumor treatment. For example, integrating the green fluorescent protein (GFP) genes into the genome of the tumor cells allows not only the observation of tumor metastasis by the fluorescence expression but also the detection at the single cell level [15]. These can simplify the histopathological procedure. As we all know, surgical resection of tumors often requires imaging guidance to provide information on tumor tissue margins, metastases, and so on. The application of fluorescence imaging-guided tumor surgery could date back to 1948. However, due to the limited local concentration and rate of tumor cell uptake of fluorescent substances in the tumor, the fluorescent imaging efficiency was weakened. In order to solve this problem, Sakuda et al. [16]designed a virus transfection system containing vesicular stomatitis virus (VSV) carrying plasmid-encoded near-infrared (NIR) fluorescent protein Katushka (rVSV-K). Katushka has the NIR wavelength ranges with excitation and emission spectra peaking at 588 and 635 nm, respectively, and is able to penetrate for several millimeters. After the viral transfection system was injected into osteosarcoma in mice, the tumor was surgically removed with the guidance of fluorescent imaging. It was proved that, compared to the traditional surgical mode, rVSV-K selectively infects osteosarcoma cells in vitro, and NIR fluorescence bioimaging using rVSV-K enables easy determination of primary tumor boundaries and resection of the tumor.

Fluorescent proteins not only play an important role in tumor surgical resection but also have a great influence in detecting tumor growth and metastasis. GFP was also used for angiogenesis monitoring and quantification, which can provide a better chance for the detection of tumor growth and metastasis *in vivo*. The protease matriptase as a type II membrane anchored-serine protease is a key factor contributing to tumor growth and metastasis. Mitchell et al. [17] developed a red fluorescent protein (ddRFP) reporter system (ex/em: 535 nm/605 nm). DdRFP systems rely on the interaction of two fluorescent protein domains, and when they bind to form a heterodimer, the fluorescence increases. Otherwise, it weakens. In this system, matripase plays a regulatory role; when the matriptase is excessively expressed, it can damage protein domains of RFP and make its fluorescence quenched, which suggests aggressive tumor growth. By designing a switch-type fluorescent probe, the growth and metastasis of tumors can be intuitively evaluated according to the fluorescence generation. This strategy makes fluorescent imaging in tumors more flexible. However, some scholars have pointed out that the fluorescence generated by GFP was dim, so it was difficult to detect or amplify the fluorescence signals, which limits the accurate detection of the target in real-time.

#### 2.1.2. Bioluminescence Imaging

Compared with fluorescence imaging, bioluminescence imaging (BLI) does not require laser radiation, and luciferase can activate bioluminescence signal generation via the activation of specific substrates directly and corresponding cofactors, which avoids the problems of phototoxicity and absorption or scattering of laser, which make BLI possess the advantage of extreme sensitivity and simple. The spectra peak at the range of luciferase is generally between 400 and 620 nm [18]. There are three main types of luciferase that are most commonly used in tumor imaging, including firefly luciferase and click beetle luciferases, the Renilla and Gaussia luciferases, and bacterial luciferases [13].

Traditional luciferase can maintain a bioluminescence signal for 10–20 minutes in the tumor, which increases imaging repeatability and reduces operational complexity. However, traditional luciferases still face some challenges in tumor imaging. The imaging of traditional luciferase is still affected in tissue penetration by other external conditions. For example, imaging signals are susceptible to basic intracellular metabolic changes, and imaging brightness is limited in deep tissue. Therefore, developing a novel luciferase reporter gene for tumor imaging is crucial for efficient tumor imaging. Coralie et al. isolated a novel luciferase from the deep sea shrimp, which was named NanoLuc. Compared to traditional bioluminescence imaging probes, such as Fluc and Rluc, NanoLuc with greater chemical stability, lower background autoluminescence, and higher photon yield were tested in glioblastoma cell lines and tumors. Due to NanoLuc possessing the advantage of high brightness, it was more suitable for deep tumor bioluminescence imaging *in vivo* [19]. In addition, NanoLuc has different substrates from firefly luciferase, so that it can be combined with Fluc for sequence detection, enabling efficient dual-report subimaging, which makes it possible to apply them to realize multicellular events in one imaging process [20].

Although BIL avoids scattering of laser, part of the signal of activated luciferase is still absorbed and scattered by tissues, which weakened the sensitivity and resolution of images [21]. To address this, Mezzanotte et al. engineered a human hepatoblastoma cell line (HepG2) with a reporter gene expressing red-shifted thermostable luciferase. The green bioluminescent signal was 75±8% absorbed, but only 20±6% absorption of the red signal in xenograft models of liver cancer. The results showed that compared to wild-type green luciferase, red-shifted fluorescence can reduce the absorption and scattering of imaging signals by tissues and skin, resulting in better imaging specificity [22]. Moreover, the researchers applied two reporter genes simultaneously to reflect two separate physiological events in a single image, which further widen the application of bioluminescence imaging technology.

The continuous improvement and optimization of luciferase probes can enhance the sensitivity of molecular tumor imaging, which provides great support for detecting the mechanism of protein-protein interaction and ligand-receptor interaction. Luciferase-based reporter systems have been used to visualize the expression of the tumor-related gene [23, 24]. CXCL12 is a kind of tumor chemokine and plays an important role in tumor growth and metastasis. [25]. Luker et al. developed a new dual luciferase imaging system, in which CXCL12 is fused to Gaussia luciferase (CXCL12-GL), utilizing the luciferase gene to track the expression level of CXCL12. In addition, firefly luciferase was used to mark the total number of breast cancer cells. The correlation between CXCL12 and CXCR7 in tumors was analyzed by fluorescence ratio (SERUM GL/tumor FL). According to the results, they successfully realize monitoring the process of chemokine scavenging by CXCR7 through dual luciferase imaging and quantify the effect of CXCR7 on tumor growth and metastasis of CXCR4-expressing breast cancer cells, which provides a useful imaging method for quantification the role of tumor chemokines and evaluation of tumor development.

#### 2.1.3. Photoacoustic Imaging

Photoacoustic (PA) tomography technology opens a new window of biomedical imaging, using a combination of optics excitation and acoustics detection to overcome the traditional depth limitations of optical imaging. PA probes with the advantages of strong penetration, high spatial resolution, and no ionizing radiation are suitable to precisely monitor physiological and pathological processes *in vivo*. Fluorescent proteins as photoacoustic imaging probes are common for tumor imaging. However, the fluorescent proteins with the low thermal conversion efficiency limit the generation of PA signal, which is a disadvantage of the amplification for the interest area. Ogunlade et al. engineered crimson fluorescent protein (FP) of E2 to change it to a darkened GFP-like protein reporter, which can produce high PA signal. The FP protein or GFP-like protein expressed by tumor cells was injected into mice, resulting in the PA signal intensity of GFP-like protein being three times than that of FP protein *in vivo* [26]. This is the first time that GFP-like proteins as PA probes are used in mammalian tissue, and the development of this novel gene probe is expected to help further photoacoustic imaging probes. Recently, many developments of genetically encoded PA probes have been demonstrated prospects in oncology applications. Based on the above, PA imaging has overcome the limitation of penetration depth and spatial resolution, which provides a powerful tool for the detection of cell fate and molecular function in deep tissues of organisms.

### 2.2. Ultrasound Imaging

Although optical imaging is the most common molecular imaging method, poor penetration of lasers limits its application. Compared with optical imaging, US enables visualization of deep tissues up to centimeter grade, with great spatial and temporal resolution (∼100 *μ*m and ∼1 ms, respectively) [27, 28]. According to the difference in the signal of ultrasonic echo waves, introducing contrast agents, such as the lipid or protein shells containing gas microbubbles, demonstrated encouraging tumor angiography [28–30]. However, the size of microbubbles is ill-suited to penetrate the vascular endothelial cell gap, which limits the efficiency of ultrasound imaging in tumors [31]. Moreover, due to the poor stability and short half-life *in vivo*, the efficiency of gas-filled microbubbles in monitoring tumors in real-time is unsatisfactory. With the rapid development of synthetic biology, genetically encoded molecular imaging probes as a novel molecular imaging tool have been researched in ultrasound imaging.

Gas vesicles (GVs) were genetically encoded from acoustic reporter genes (ARGs), which are composed of the structural protein gene GvpA and GvpC from *A. flos-aquae* and the assembly factor gene from *B. megaterium* [32]. GVs are nanoscale imaging probes, about 200 nm in size and 2 nm in shell thickness, whose shells are composed of amphiphilic protein structures that allow gas exchange from the surrounding medium to the hollow interior, but exclude the aqueous phase. Due to this special structure, GVs were more stable and had a longer half-life than chemosynthetic ultrasound contrast agents *in vivo*. Shapiro et al. [33, 34]designed the engineered bacteria, integrating ARG1 and luminescence operon luxABCDE (Lux), and injected them into the central or marginal region of colon cancer to evaluate the performance of ultrasound imaging in tumor monitoring. The results showed that ultrasound imaging could more clearly display the specific distribution of bacteria in the tumor, which realized the spatial localization of deep tumors. This strategy provides a more indepth and intuitive monitoring tool for mammalian microbiome interactions and facilitates the development of diagnostic and therapeutic agents.

The previously mentioned method uses bacteria to produce gas vesicles for indirectly in tumor imaging via the target function of bacteria. Furthermore, infecting genes into tumor cells make cells express gas vesicles directly, which can show cells' growth and metastasis more intuitively, especially cellular processes occurring inside intact organisms. It is necessary to develop an acoustic reporter genes expression system from prokaryotes to eukaryotes. In 2019, Shapiro et al. [35] continued their previous work involving ARG and GVs and made a major breakthrough. The research group designed a eukaryotic genetic program based on the bacterial ARG gene cluster and introduced it into mammalian cells, which enhanced the ultrasound contrast signal of transfection cells due to the GVs production. It was proved that mammalian acoustic reporter genes allow cells to be visualized at volumetric densities below 0.5%. Furthermore, in order to evaluate the ultrasound imaging efficiency of ARG engineered mammalian cells *in vivo*, the research group introduced the ARG gene into HEK-293T and inject them subcutaneously into the flank of the mice. It was shown that the pattern of gene expression persists in tumors, the structure of tumor tissue could be observed clearly by ultrasound, and the distribution of ultrasound signal was consistent with pathological tissue sections of the tumor, which showed the application potential of ARG in monitoring tumor cells *in vivo*.

### 2.3. Magnetic Resonance Imaging

Compared with the other imaging mode, magnetic resonance imaging (MRI) is a high-resolution imaging method with good tissue contrast that is not affected by depth [36]. However, due to the disadvantage of low sensitivity in MRI imaging, MRI contrast agents are particularly important in order to improve the contrast between tumor tissue and normal tissue. MRI contrast agents, such as Gd-DTPA, could change the relaxation rate of water particles in the interest region and improve the tissue contrast and imaging quality through the enhanced signal. Although MRI contrast agents have been widely applied in clinical practice, there still remains limitation on specificity, accuracy, and even biosafety. Recently, FDA published public health warning on Gd contrast agents, which mentioned that Gd contrast agents may induce nephrogenic systemic fibrosis or nephrogenic fibrosing dermopathy.

Compared with MRI contrast agents, genetically encoded reporters have good biocompatibility, and they can image at the cellular and molecular level, visualizing the expression and activity of genes, proteins, and cells [37–40]. In addition, therapeutic response efficiency can be quantified via the detection of genetically encoded reporters' expression, whose signals were generated by gene or protein expression. For example, overexpressed metalloproteins and metal ion transporters will enrich the paramagnetic content of cells and enhance the nuclear relaxation rates, thereby enhancing contrast in *T*_1_ or *T*_2_ weighted MR [41, 42]. In the next part, we will briefly introduce some typical examples of genetically encoded molecular imaging probes for MRI in tumor imaging.

Generally, iron is absorbed in many tissues and cells through the classical transferrin (Tf) and transferrin receptor pathways. Ferric iron first binds to Tf and then binds to TfR on the cell surface. After the consecutive processes of endocytosis, acidification, release, and migration, iron enters the cytoplasm and performs its biological function. It has been proved that TfR was overexpressed in cells with a high rate of proliferation, especially in tumor cells [43, 44]. Therefore, the overexpression of TfR can improve iron uptake, which decreases T2 relaxation time, enhancing the MRI imaging signal of the tumor area [45].

Compared with TfR, the action mechanism of the tyrosinase-melanin system (TYR) is simpler in MRI imaging. The system uses tyrosinase to catalyze the synthesis of melanin, and the synthesized melanin chelates with metal ions efficiently, thus shortening the T1 relaxation time of metal ions, resulting in a high characteristic signal on T1-weighted images [46]. Despite the ability of chelating metal, melanin also has the advantage of a broad optical absorption spectrum and easy decoration with chemical probes, which make TYR the ideal reporter genes to realize multimodality molecular imaging. Based on these, Qin et al. [47] built breast cancer cells that could express TYR via introduced plasmids that encode TYR into MCF-7 cells by gene transfection. TYR reporter expressed tyrosinase then catalyzes the tyrosine precursor to synthesize melanin. Melanin has the ability to chelate metal ions (Fe^3+^) which provides contrast for MRI, and the characteristic of a broad optical absorption spectrum is suitable for PAI. Moreover, melanin can be specifically subjected to chemical modification by 18F–P3BZA for PET. It is proved that the growth of breast tumors could be monitored under photoacoustic/MR/PET imaging, which provided more diverse imaging information for tumor detection. However, some studies also indicated that overexpression of melanin could impair cells. In order to reduce the risk of nonspecific side effects of melanin, controlled expression means that the expression rate of TYR should be controlled [48]. Therefore, Alfke et al. designed a plasmid consisting of a tetracycline-controlled transactivator and TYR gene. With the control of tetracycline and doxycycline separately, the expression of TYR gene showed an excellent on-off effect [49], which provides a potential safety strategy and shows the potential to reduce background signal and enhance imaging specificity for tumor imaging.

MRI reporter genes mentioned above, such as metalloproteinase and metal iron receptor, still had their limitation of their reliance on metals or relatively low sensitivity. Thus, some novel nonmetallic reporters were developed for MRI imaging, such as aquaporin(AQP), which were proteins that transport water molecules across membranes [50]. When it is overexpressed, water transport would increase, which can also generate an MRI signal [51]. The occurrence and development of the tumor is closely related to the diffusion process of water transport. Not only that, based on the clinical case and histogram analysis, it has been proved that the expression level of AQP in tumor tissue, including ovarian cancer and prostate cancer, has a strong relationship with the b-value diffusion MRI signal, which also suggested that AQP-based MRI provided a novel noninvasive mode for predicting the level of malignancy of tumor [52, 53].

### 2.4. Nuclear Medicine Imaging

Nuclear medicine imaging mainly includes single photon emission computed tomography (SPECT) and positron emission tomography (PET). Combined genetically encoded molecular imaging probes with nuclear medicine tomography are widely used in tumor imaging, mainly including tracking cell levels, monitoring cancer progression and metastasis, and evaluating the efficacy of anticancer therapy. For example, the herpes simplex virus type 1 thymidine kinase (HSV1-TK) genetic sequence was designed to selectively uptake 18F to locate and track therapeutic substances in glioma [54].

Among radionuclide gene probes, sodium iodide symporter (NIS) is considered one of the most valuable in preclinical and translational studies, which has been widely used in the diagnosis and treatment of tumors. NIS is usually expressed in thyroid follicular cells and can mediate the uptake of iodide ions. Zhang et al. designed oncolytic vesicular stomatitis virus (VSV) to encode NIS, via mediating the uptake of 125I to realize radionuclide imaging. It can noninvasively monitor pharmacokinetic activity and viral invasion of tumors when visualized by single photon emission computed tomography (SPECT/CT). At the same time, they accurately measured the extent of virus-mediated cell killing and oncolytic potency by using 99mTc neomycin as a radioactive tracer [55]. However, serval scientists found that overexpression of NIS in the early stage will affect the function of the recombinant virus [56]. Therefore, it is necessary to find appropriate strategies to regulate NIS expression for tumor imaging. Wang et al. engineered a synthetic promoter for the regulation of NIS expression, which increased protein expression and 123I or 99Tc uptake [57], thus improving effectively centralized PET/SPECT tracers to facilitate widespread use in preclinical imaging.

## 3. Limitation

The design and application of molecular imaging probes based on biosynthesis involve many theories, methods, and techniques. Although it has a wide range of applications, there are still limitations in this field. Some methods of application of gene synthesis probes involved gene transfection. Obviously, selecting appropriate methods for effective transfection of exogenous genes is the key for gene transfection.

At present, viruses were used as vectors as the most common and effective method which has a high transfection rate and excellent tumor targeting [58]. When virus vectors are used for transfection in in vitro, the transfection rate can reach 100%. They generally integrate foreign genes into chromosomes by infecting specific host cells. However, it raises many safety concerns such as the interference of viral genes, cytotoxicity, and immunogenicity, especially transfected in vivo. The emergence of nonviral vectors including liposomes or lipid complexes, cationic polymer, nanocarriers, etc., (noninfectious) provide solutions to strengthen security in *in vivo* [59, 60].At present, cationic liposomes and cationic polymer-mediated have been used for gene transfection *in vivo* [60]. Previously, we carried out research on the physical delivery gene transfection mode, using the cavitation effect of ultrasound to carry out gene-targeted transfection. Ultrasound, as a noninvasive control method, can reach the deep tissue at a fixed point, which can solve the passive diffusion of nonviral vectors while ensuring safety [61]. However, most nonviral methods are less efficient than viral methods for gene transfer. Therefore, how to get an ideal transfection method with high efficiency and minimal toxicity is the key to the study [62].

## 4. Prospect and Conclusion

Molecular imaging contributes to our understanding of the growth and development of tumors at more microscopic cellular and molecular function levels [10]. In contrast to chemicals, genetically encoded molecular imaging probes can real-time and long-acting monitor specific cells or proteins of interest in tumor tissues and have higher biological compatibility, stability, and tissue contrast *in vivo*. Therefore, it has attracted increasing attention from researchers in engineering and biomedicine.

At present, researchers focus more on how to improve the imaging effect of the gene reporters, which generally reflects the cell level of the tumor. However, the application of gene reporters for imaging molecular biological events such as tumor gene and molecular level has not been studied in depth. What should be focused next is the application in tumor imaging. These proven and mature imaging systems are really used to reflect the molecular biological events in tumors, which can realize real-time monitoring through the imaging system. Molecular imaging of gene synthesis has a good application prospect in tumor diagnosis and mechanism exploration.

In summary, genetically encoded imaging reporters will be designed for high sensitivity, spatial resolution, and biocompatibility. These reporters may prove invaluable for understanding intercellular communications, yielding a better fundamental understanding of complex biologic systems that hopefully will in turn yield better cancer diagnostics and therapeutics [36].

## Figures and Tables

**Figure 1:** Application of genetically encoded molecular imaging probes in tumor imaging.

## Abbreviations

MRI: Magnetic resonance imaging
GVs: Gas vesicles
ARGs: Acoustic reporter genes
GFP: Green fluorescence protein
Tf: Transferrin
TYR: Tyrosinase-melanin system
AQP: Aquaporin
VSV: Vesicular stomatitis virus
RFP: Red fluorescent protein
PET: Positron emission tomography
SPECT: Single photon emission computed tomography
HSV1-TK: Herpes simplex virus type 1 thymidine kinase
PA: Photoacoustic
FP: Fluorescent protein.

## Additional Points

With the development of interdisciplinary science, imaging technology has entered a fast lane in recent years. Molecular imaging is recognized as the most promising imaging technology in the 21^st^ century, and molecular imaging probes play key role in it. With the application of chemosynthetic molecular imaging probes in the clinic, the safety and stability of probes have been widely concerned. Synthetic biology provides an important strategy for this problem. Genetically encoded molecular imaging probes have significant advantages in sensitivity, stability, and biocompatibility. In this review, we will focus on the application of gene-encoded molecular imaging probes in tumor diagnosis.
